This article has been retracted.

# Evaluating the Anticancer Activity of Blocking TNF Type 1 Receptors in Thioacetamide-Induced Hepatocellular Carcinoma in a Rat Model

**DOI:** 10.7759/cureus.32519

**Published:** 2022-12-14

**Authors:** Alaa Bagalagel, Reem Diri, Ahmed Noor, Deina Almasri, Hussain Bakhsh, Hussam I Kutbi, Mohammed M Al-Gayyar

**Affiliations:** 1 Clinical Pharmacy, King Abdulaziz University Faculty of Pharmacy, Jeddah, SAU; 2 Clinical Pharmacy, King Abdulaziz University, Jeddah, SAU; 3 Pharmacy, King Abdulaziz University, Jeddah, SAU; 4 Pharmaceutical Chemistry, University of Tabuk Faculty of Pharmacy, Tabuk, SAU; 5 Biochemistry, Mansoura University Faculty of Pharmacy, Mansoura, EGY

**Keywords:** heme oxygenase-1 (ho-1), hepatocellular carcinoma (hcc), nuclear factor erythroid 2-related factor 2 (nrf2), tnf-α type 1 receptor (tnfr1), tumor necrosis factor (tnf)-α

## Abstract

Background

Hepatocellular carcinoma (HCC) can explicate about 90% of the total primary liver cancer cases, with approximately 800,000 new cases identified each year worldwide. In addition, any changes in the expression of the tumor necrosis factor α (TNF-α) type 1 receptor (TNFR1) might impact many biological processes, which may lead to cancer.

Aims

We conducted the following study to investigate the ability of CAY10500, a TNF-α inhibitor that prevents binding to the TNF receptor 1, to produce anticancer effects against hepatocellular carcinoma experimentally induced in rats and to discover its effect on nuclear factor erythroid 2-related factor 2 (Nrf2) and heme oxygenase-1 (HO-1).

Materials and methods

HCC was induced in rats via 200 mg/kg thioacetamide followed by treating some rats with IV 1 mg/kg CAY10500. Assessment of the liver impairment was by measuring the serum α-fetoprotein (AFP) and investigation of liver sections stained with hematoxylin/eosin. The hepatic expression of both the messenger RNA (mRNA) and protein levels of TNF-α, TNFR1, Nrf2, and HO-1 was assessed.

Results

We found that CAY10500 increased the survival percent of rats associated with a reduction in serum AFP and the number of hepatic nodules. Besides, CAY10500 reduced the expression of TNFR1 without affecting the expression of TNF-α. Finally, CAY10500 increased the expression of both Nrf2 and HO-1.

Conclusions

Inhibition of TNFR1 expression in HCC by using CAY10500 produced therapeutic effects as indicated by increasing the survival rate, reducing the serum AFP level, decreasing liver nodules, and improving hepatocytes’ structure. In addition, TNFR1 significantly enhanced the expression of Nrf2 and HO-1.

## Introduction

Hepatocellular carcinoma (HCC) represented 90% of the primary liver cancer with increased global spread annually, as it is responsible for 800,000 new cases worldwide [1]. Several signaling pathways were linked with the pathogenicity of HCC such as growth factors, cell differentiation, and angiogenesis [2]. Although there are many advances in HCC discoveries, there are just a few effective treatment options for HCC patients [3]. Furthermore, because of the strong angioinvasive capability of the tumor, the therapeutic alternatives for HCC patients are limited [4]. Therefore, HCC is linked to a high rate of mortality and a poor prognosis [5]. Only the early stages of the disease are curative through liver transplantation (LT) and surgical resection [6]. In advanced cases, the strong angioinvasive capability of the tumor limits the therapeutic alternatives [4]. Therefore, as many cases were discovered at a late stage upon diagnosis, resistance to existing therapy and a high likelihood of recurrence leads to about an 18% five-year total survival rate for HCC patients [7].

Tumor necrosis factor (TNF)-α is a pro-inflammatory cytokine with a great role in both the initiation and propagation of inflammation and immunity [8]. After stimulation, the biological actions of TNF-α take place via two receptors, TNFRp55 (TNFR1) and TNFRp75 (TNFR2) [9]. TNFR1 is the primary signaling receptor for the host immune response and the pro-inflammatory and cytotoxic effects of TNF [10].

TNFR1 is associated with both the development and progression of many cancers such as HCC [11]. In HCC, TNFR1 is essential in the growth of oval cells during the preneoplastic stage of liver carcinogenesis. In parallel, any loss of activity of TNFR1 inhibits the incidence of tumors [12]. Therefore, many efforts have been made to target TNF-α or TNFR1 in various malignancies with pharmaceuticals that include TNF-α inhibitors, TNFR1 monoclonal antibodies, and TNFR1-targeting nanomaterials [11]. We have previously published research about using QNZ, an inhibitor of both TNF-α and NFκB, to treat experimentally induced HCC in rats. QNZ significantly reduced the expression of inflammation, oxidative stress, and fibrosis [13]. Therefore, the next step will be to evaluate the ability to block TNFR1 receptors in treating HCC. Therefore, we aimed to use CAY10500, a TNFα inhibitor that prevents binding to TNFR1, as a potential therapeutic agent against experimentally induced HCC in rats. In addition, we aimed to investigate its effect on the expression of both heme oxygenase-1 (HO-1) and nuclear factor erythroid 2-related factor 2 (Nrf2).

## Materials and methods

Animals

All animal methods were conducted in accordance with relative guidelines and approved by the Ethical Committee of the University of Tabuk under number UT-42-3-2018. Forty male Sprague Dawley rats weighing 150-200 g and aged 8-10 weeks old were used. Rats were housed in stainless-steel cages under standard housing conditions, a temperature of 25±1⁰C, with 12h light and dark cycles. The rats were divided into four groups with 10 rats each. The control group rats were injected with normal saline for 16 weeks on a daily basis. CAY10500 treated control group rats were given 1 mg/kg CAY10500 (Santa Cruz Biotechnology Inc, Dallas, Texas) via intravenous injection (IV) twice a week for 16 weeks. The HCC group rats were given 200 mg/kg via intraperitoneal injection (IP) of thioacetamide in normal saline twice weekly for 16 weeks. Finally, the CAY10500-treated HCC group rats were administered 200 mg/kg (IP) thioacetamide in normal saline twice weekly accompanied by 1 mg/kg IV CAY10500 twice weekly for 16 weeks.

Sample collection

Thiopental sodium (40 mg/kg, i.p.) was used to anesthetize rats. Serum specimens were centrifuged at 3000 rpm for 5 min after being collected from the retro-orbital plexus. Serum samples were stored at -80⁰C. A portion of the hepatic loop was separated, sliced, and kept in a 10 % buffered formalin solution followed by investigating morphological features. Another portion of the hepatic loop was homogenized in a 10-fold volume phosphate buffer of pH 7.4 and stored at -80⁰C.

Histopathological examination

Hepatic slices that are kept in 10% formalin were embedded in paraffin blocks and cut at 5 mm thickness. Sections were anonymously coded and examined in a masked manner. For immunohistochemistry, sections were incubated with monoclonal anti-Nrf2 (Sigma Aldrich Chemicals Co., St. Louis, Missouri) at 4⁰C. Sections were then incubated with the horseradish peroxidase-conjugated antibody. Next, 2% of 3,3′-diaminobenzidine in Tris-buffer was used as a chromogen. Hematoxylin was used as a counterstain.

Enzyme-linked immunosorbent assays (ELISA) determination

Commercially available ELISA kits were used for the assessment of α-fetoprotein (AFP), TNF-α (USCN Life Science Inc. Houston, TX), TNFR1 (Abcam Co, Boston, MA), and Nrf2 and HO-1 (MyBioSource, Inc. San Diego, CA) according to the instructions of the manufacturer.

Quantitative real-time polymerase chain reaction (RT-PCR)

The gene expression of TNF-α, TNFR1, Nrf2, and HO-1 mRNA levels in rat liver lysate was performed as described previously by our group [13-15]. GAPDH was used as a housekeeping gene and internal reference control. The gene-specific PCR primers used were summarized in Table 1.

**Table 1:** Primer sequences for a real-time PCR assay HO-1, heme oxygenase-1; Nrf2, nuclear factor erythroid 2-related factor 2; TNF-α, tumor necrosis factor-α; TNFR1, TNF-α type 1 receptor

Gene	Primer pair sequences	Gene ID
TNF-α	F: 5`-AAATGGGCTCCCTCTCATCAGTTC-3`	X66539
	R: 5`-TCTGCTTGGTGGTTTGCTACGAC-3`	
TNFR1	F: 5`-CCAAGTGCCACAAAGGAACC-3`	NM_013091.2
	R: 5`-TCAGGTAGCGCTGGAATTGG-3`	
Nrf2	F: 5`-AGCAGGACATGGATTTGATT-3`	XM_032903520.1
	R: 5`-CTTCTCCTGTTCCTTCTGGA-3`	
HO-1	F: 5`-ACAGAAGAGGCTAAGACCG-3`	XM_032887931.1
	R: 5`-CAGGCATCTCCTTCCATT-3`	
GAPDH	F: 5′-CCATCAACGACCCCTTCATT-3′	NM_017008
	R: 5′-CACGACATACTCAGCACCAGC-3′	

Statistical analysis

The results were presented as mean ± SEM. The normality of the distribution of samples in the study was examined using the Kolmogorov-Smirnov test. For checking rat survival, the Kaplan-Meier procedure was used. For determining significant differences among groups, one-way analysis of variance (ANOVA) was used then followed by the Bonferroni post hoc test. SPSS version 20 (IBM Corp., Armonk, NY) was used for the assessment of the statistical analysis. P < 0.05 was considered to indicate a statistically significant difference.

## Results

Effect of CAY10500 on the expression of TNF-α and TNFR1

The HCC group showed a significant increase in both mRNA and protein levels of the hepatic TNF-α and TNFR1. CAY10500 did not affect the gene and protein expression of TNF-α while it succeeded to restore gene and protein expression of TNFR1 to the basal levels In the HCC group without affecting the control group (Figure 1).

**Figure 1:** Effect of 1 mg/kg CAY10500 on hepatic gene expression of tumor necrosis factor (TNF)-α (a) and TNF type 1 receptor (TNFR1, c) as well as protein expression of TNF-α (b) and TNFR1 (d) * Significant difference as compared with the control group at p<0.05. # Significant difference as compared with the HCC group at p<0.05 HCC, hepatocellular carcinoma; TNF-α, tumor necrosis factor-α; TNFR1, TNF-α type 1 receptor

Effect of CAY10500 on survival rate in a rat model

The HCC group had a reduced survival percentage by about 70% compared to the control group. The treatment of HCC rats with CAY10500 increased the survival percent of rats to 80% as compared to the control group (Figure 2a).

**Figure 2:** Effect of 1 mg/kg CAY10500 on rats’ survival (a), the average number of nodules (b), and serum AFP (c) * Significant difference as compared with the control group at p<0.05. # Significant difference as compared with the HCC group at p<0.05. AFP, alpha-fetoprotein; HCC, hepatocellular carcinoma

Effect of CAY10500 on the number of hepatic nodules and serum AFP tumor marker

HCC showed a significant elevation in the number of hepatic nodules compared with the control group associated with a significant increase in the serum level of AFP. CAY10500 treatment results in a 65% reduction in the number of hepatic nodules and a 60% reduction in the serum level of AFP in the HCC group without affecting the control group (Figures 2b-2c).

Effect of CAY10500 on the histology of liver tissue

Microscopic pictures of liver sections from the control group stained with H&E showed normally arranged hepatic cords around central veins. A liver section from the HCC bearing group shows well‐differentiated HCC. Cells of HCC are polygonal with distinct cell membranes, eosinophilic granular cytoplasm, and hepatocytes showing vacuolar to ballooning degeneration (yellow arrows). Sections from the HCC group treated with 1 mg/kg CAY10500 reduced the degeneration of hepatocytes. In addition, an investigation of the mitotic score revealed a 69% reduction in HCC rats treated with CAY10500 as compared with the HCC group without affecting the control group (Figure 3).

**Figure 3:** Hepatic sections stained with hematoxylin and eosin in the control group (a), control group treated with CAY10500 (b), hepatocellular carcinoma (a), and hepatocellular carcinoma treated with CAY10500 (d), as well as mitotic score (e) Yellow arrows represented hepatocytes showing vacuolar to ballooning degeneration. Black arrows represented mild regression of hepatic fibrosis. * Significant difference as compared with the control group at p<0.05. # Significant difference as compared with the HCC group at p<0.05. The scale bar represented 50 µm. HCC, hepatocellular carcinoma

Effect of CAY10500 on both mRNA and protein levels of Nrf2

The HCC group showed a 55% increase in both mRNA and protein levels of hepatic Nrf2 when compared to the control group. CAY10500 succeeded to restore both its mRNA and protein to the normal levels as the control group in the HCC group without affecting the control. A parallel investigation of hepatic sections stained with anti-Nrf2 antibodies revealed a reduction in the immunostaining in the sections from the HCC group, which was reversed by treatment with CAY10500 (Figure 4).

**Figure 4:** Effect of 1 mg/kg CAY10500 on hepatic gene expression of nuclear factor erythroid 2-related factor 2 (Nrf2, a) and its hepatic protein level (b). Hepatic sections stained with anti-Nrf2 antibodies in the control group (c), control group treated with CAY10500, HCC group (e), and HCC treated with CAY10500 (f) * Significant difference as compared with the control group at p<0.05. # Significant difference as compared with the HCC group at p<0.05. Scale bar 100 μm. HCC, hepatocellular carcinoma

Effect of CAY10500 on both the mRNA and protein levels of HO-1

The HCC group showed significantly elevated levels of both mRNA and protein of hepatic HO-1 as compared to the control group. CAY10500 reduced the elevated both mRNA and protein levels of hepatic HO-1 in the HCC group without affecting the control group (Figure 5).

**Figure 5:** Effect of 1 mg/kg CAY10500 on the hepatic gene expression of HO-1 (a) and its hepatic protein level (b) * Significant difference as compared with the control group at p<0.05. # Significant difference as compared with the HCC group at p<0.05. HCC, hepatocellular carcinoma; HO-1, heme oxygenase-1

## Discussion

HCC is the sixth most widespread cancer and the fourth most worldwide cause of cancer-related death. There are many systemic drugs approved by the Food and Drug Administration (FDA) for advanced HCC treatment. The current guidelines' treatment suggestions for advanced-stage HCC include the atezolizumab and bevacizumab combination as the preferred regimen for Child-Pugh A patients; sorafenib, lenvatinib, and immunotherapy are other options [16]. Although the most effective treatment of patients with early clinical stage is liver resection and transplantation, these techniques are not suitable for most patients. Therefore, HCC is placed as the second most lethal cancer, with a five-year survival of about 18% [1].

Infiltration of immune cells in the HCC microenvironment has a great role in tumor cell initiation, growth, and metastasis. The activation of immune cells leads to the production of pro-inflammatory and immune-stimulatory cytokines such as TNF-α, INF-β1, and interleukins. HCC is characterized by a great elevation in the expression of many genes [17]. The translocation of NFκB followed by stimulation of TNF-α as a downstream pathway controls cellular inflammation and proliferation with subsequent progression of HCC [18]. Moreover, inflammatory cytokines such as TNF-α are highly elevated in HCC patients [19]. We have previously shown that the inhibition of both TNF-α and NFκB significantly had therapeutic effects against HCC in rats [13]. Therefore, we used CAY10500, a TNFα inhibitor that prevents binding to TNFR1, in the current study. In addition, the pathogenicity of HCC is linked to an inflammatory response in patients. We found that CAY10500 inhibits the expression of TNFR1 without affecting the expression of TNF-α in HCC rats without affecting the control rats. In addition, we have found that treating HCC rats with CAY10500 significantly increased rats’ survival, reduced the number of nodules per nodule-bearing liver, reduced serum AFP levels, and was associated with improvement in the structure of hepatocytes and reduction of the mitotic score. CAY10500 was not used previously in the treatment of HCC.

Oxidative stress is considered a major player in both the development and progression of HCC by affecting cell proliferation, apoptosis, and cell cycle [20,21]. When the status of oxidative stress begins, reactive oxygen species (ROS) showed a detrimental effect on many body cells, leading to the progression of chronic liver disease and hepatocarcinogenesis. Interestingly, ROS are activators of autophagy and many stress response molecules as nuclear factor (erythroid-derived 2)-like 2 (Nrf2) [22]. Aggregation of cytoplasmic Nrf2 activates nuclear migration and enhances the transcription of antioxidant and detoxification agents that promote cellular protective response toward oxidative stress [23]. In parallel, the deactivation of Nrf2 was related to the progression of HCC, including metastasis [24]. In addition, inhibition of Nrf2 significantly enhanced the erastin- and sorafenib-induced suppression of HCC [25]. One of the downstream of Nrf-2 is HO-1, which is one of the antioxidant defense proteins [26,27]. HO-1 overexpression participates in the pathogenesis and progression of some malignancies. In addition, HO-1 activation is considered cytoprotection [28]. We found that CAY10500 reversed the HCC-induced reduction in the expression of Nrf2 and HO-1. However, no previous study illustrated the effect of CAY10500 on the expression of both Nrf2 and HO-1 in HCC models.

The mechanism of action of CAY10500 is summarized in Figure 6. 

**Figure 6:** Schematic presentation of the protective effects of CAY10500 in HCC HO-1, heme oxygenase-1; HCC, hepatocellular carcinoma; Nrf2, nuclear factor erythroid 2-related factor 2; TNF-α, tumor necrosis factor-α; TNFR1, TNF-α type 1 receptor

There are some limitations in the study, as rats have different metabolic pathways and drug metabolites than humans, leading to different dosing and various ways of the body dealing with the drugs. In addition, there are many methods for tumor induction in rats; we only used the chemical induction of HCC in rats using thioacetamide.

## Conclusions

The inhibition of TNFR1 expression in HCC by using CAY10500 produced therapeutic effects as indicated by increasing the survival rate, reducing serum AFP level, decreasing liver nodules, and improving hepatocytes’ structure. In addition, TNFR1 significantly enhanced the expression of Nrf2 and HO-1. The work opens a new window to treating HCC by modulating TNFR1. Finally, more work is needed to illustrate the mechanism of action and to use other substances with the ability to inhibit TNFR1.
